The article "L-securinine inhibits cell growth and metastasis of human androgen-independent prostate cancer DU145 cells via regulating mitochondrial and AGTR1/MEK/ERK/STAT3/PAX2 apoptotic pathways" was published in 2019. Journal: Biosci Rep.

# L-securinine inhibits cell growth and metastasis of human androgen-independent prostate cancer DU145 cells via regulating mitochondrial and AGTR1/MEK/ERK/STAT3/PAX2 apoptotic pathways

**DOI:** 10.1042/BSR20190469

**Published:** 2019-05-10

**Authors:** Dongxu Zhang, Houxian Liu, Binbin Yang, Jiasheng Hu, Yue Cheng

**Affiliations:** 1 Department of Urological Surgery, Ningbo First Hospital, Ningbo Hospital of Zhejiang University, Ningbo 315010, China; 2 Department of Urological Surgery, Ningbo Fenghua District People’s Hospital, Ningbo 315500, China

**Keywords:** Androgen-independent prostate cancer (AIPC), Apoptosis, L-securinine, Mitochondrial apoptotic pathway

## Abstract

The present study aims to evaluate the anticancer effect of L-securinine on androgen-independent prostate cancer (AIPC) DU145 cells. L-securinine (2.5, 5, and 10 μM) treatment for 24, 48 and 72 h displayed strong growth inhibitory effect on DU145 cells in a concentration and time-dependent fashion but has less toxicity toward normal androgen-dependent LNCaP cells. Hoechst 332582 staining of DU145 cells and Annexin V-FITC/ PI dual-labeling followed by flow cytometry assay identified that this growth inhibition by L-securinine would be due to the induction of apoptosis. Moreover Transwell assay revealed that L-securinine significantly inhibited the cell migration/invasion ability of DU145 cells. Furthermore, results of western blotting showed that the involvement of mitochondrial apoptotic pathway in the L-securinine-induced apoptosis of DU145 cell, as evidenced by an increase in the protein expression of Bax, cleaved caspase-9, cleaved caspase-3, cytosolic cytochrome c, and cleaved PARP, together with a unchanged cleaved caspase-8 and decreased Bcl-2 protein expression. Also, L-securinine-induced antimetastatic activity in DU145 cells was associated with decreased protein expression of MMP-2 and MMP-9 and concurrent reduction of VEGF. In addition, further studies revealed that L-securinine may inhibit the protein expression of AGTR1, p-MEK1/2, p-ERK1/2, p-STAT3, PAX2, and p-PAX2, while the expression of ERK1/2, MEK1/2, and STAT3 protein retains intact. These findings suggest that L-securinine may be a promising chemopreventive agent against AIPC.

## Introduction

Prostate cancer continues to be one of the most prevalent malignancies, and is the second leading cause of death amongst older men in western countries such as Europe and the United States [1], while its incidence is low in Asian countries. Recently, prostate cancer has ranked as the fifth most common cancer for men in China, though it has only jumped to prominence in China over the past 10 years [2]. Although molecular mechanisms underlying onset and progression of prostate cancer are not clear, there is also a growing recognition amongst physicians that the cause of this frequently occurring disease arose mainly from a shift toward western diets and lifestyles. Another is considered to be altered gene expression in patients due to environmental factors [3]. A sharp rise in prostate cancer cases together with an increasing mortality rates has caught China’s healthcare system short-handed when it comes to making advanced surgical techniques available to all those who need it. To date, radical prostatectomy, radiotherapy, and hormonal therapy are effective options to treat localized disease at an early stage, but clinical management of advanced prostate cancers has been challenging [4]. Initially, hormone therapy for patients with advanced and aggressive prostate cancer generally achieves good efficacy with a high response rate of 80–90%, and has been the standard treatment for prostate cancer [5]. However, most patients receiving androgen ablation progress to a hormone-refractory state several years after the initial therapy, eventually making them unresponsive to further hormonal manipulation and leads to a fatal outcome in many cases [6,7]. Moreover, chemotherapy and radiation therapy are largely ineffective against advanced prostate cancer, and has serious toxic side effects [8,9]. Therefore, treatment approaches for androgen-independent prostate cancer (AIPC) are unsatisfactory and the survival of those patients remains poor. Thus, there is a strong demand to develop novel therapeutic agents to treat and prevent this advanced malignancy.

Nowadays, more and more naturally bioactive compounds found in traditional Chinese medicine have received extensive attention for cancer therapy by researchers because of their high activity and low cytotoxicity [10]. Securinine, a major plant-derived alkaloid from *Securinega suffruticosa*, exhibits a wide spectrum of biological activities, such as antimalarial and antibacterial activities [11]. Typically, modern pharmacological studies have shown that L-securinine (Figure 1), one of the optical isomers of securinine [12], plays a critical role of antitumor activity in human cancer cell lines, making it a promising candidate for the development of future cancer therapies [13–15]. Despite wide pharmacological properties associated with L-securinine, little information, if any is available in term of the antitumor effect of L-securinine on human prostate cancer cells and the underlying molecular mechanisms remain poorly understood. The present study was therefore designed to investigate the effects of L-securinine on the growth and metastasis of androgen-dependent or independent prostate cancer cells and to explore the possible mechanisms of action.

**Figure 1:** The molecular structure of L-securinine

## Materials and methods

### Materials and chemicals

MTT, fetal bovine serum (FBS), DMSO, and L-Securinine were obtained from Sigma (St. Louis, MO, U.S.A.). Anti-Bax, Bcl-2, cleaved caspase-9, cleaved caspase-8, cleaved caspase-3, cytosolic cytochrome c, cleaved PARP, MMP-9, MMP-2, AGTR1, MEK1/2, p-MEK1/2, ERK1/2, p-ERK1/2, STAT3, p-STAT3, PAX2, p-PAX2, and VEGF antibodies were obtained from Santa Cruz Biotechnology, Inc. (Santa Cruz, CA, U.S.A.). Annexin V–fluorescein isothiocyanate (FITC)/propidium iodide (PI) kit, Transwell chambers and Matrigel gel was from BD Biosciences (San Jose, CA, U.S.A.).

### Cell lines and cultures

Androgen-independent DU145 cell line and androgen-dependent LNCaP cell line were purchased from the Cell Bank of Type Culture Collection of Chinese Academy of Sciences (Shanghai, China), and were cultured in DMEM supplemented with 10% heat–inactivated FBS, penicillin (10 U/ml) and streptomycin (10 μg/ml), in a humidified incubator (Sanyo XD–101; Sanyo Electric Co., Ltd., Osaka, Japan) with 5% CO_2_ at 37°C

### MTT assay

Cell viability was assessed using MTT assay. Cells (2 × 10^5^) in a logarithmic phase were inoculated into a 96-well plate for 24 h, followed by treatment with different concentrations of L-securinine (2.5, 5, and 10 μM) for 24, 48, and 72 h. Then, 20 μl of stock solution of MTT (5 μg/ml) was added to each well, and the cultivation was continued for 4 h before the culture medium mixture was discarded. Finally, 150 μl DMSO was added to each well and gently oscillated at room temperature for 10 min. The optical density was measured with a spectrophotometer (Bio-Rad Laboratories, Hercules, CA, U.S.A.) at 470 nm wavelength. Cell viability was expressed as a percent of control group and each experiment was performed in triplicate.

### Apoptosis analysis using Hoechst 33258 staining

Hoechst 33258 staining was used to investigate the nuclear morphologic changes of apoptotic cells [16]. Briefly, after exposure to different concentrations of L-securinine (2.5, 5, and 10 μM) for 48 h, cells were washed with cold PBS and fixed with freshly prepared 4% paraformaldehyde for 15 min at room temperature. Then the fixed cells was rinsed with PBS and stained with 500 μl Hoechst 33258 solutions (10 μg/ml) in compliance with the manufacturer’s instructions. Finally, the cells were washed thrice with PBS and Hoechst 33258-stained nuclei were observed using an inverted fluorescence microscope (Olympus, BX53, Japan).

### Apoptosis analysis by flow cytometry

Annexin V-FITC/PI Apoptosis Detection Kit was used to quantitate the percentage of cells undergoing apoptosis according to the manufacturer’s instructions and performed as described previously [17]. Briefly, treated cancer cells (3 × 10^5^ cells/well) in six-well plates were collected, washed twice with ice cold PBS, centrifuged at 1000 ***g*** for 5 min, and then resuspended in 100 μl of binding buffer containing 5 μl of annexin V-FITC and 5 μl of PI in the dark at ambient temperature. After 15 min, these cells were subjected to FACScan flow cytometry (Becton & Dickinson Co., U.S.A.) to quantitate the cell apoptosis rate. Events were recorded statistically (10,000 events/sample) using CellQuest software (BD Biosciences).

### Transwell invasion and migration assay

Transwell chambers coated with or without Matrigel were used to assay the invasion and migration of prostate cancer cells *in vitro*, respectively. In brief, cells (2 × 10^4^/well) were plated into the upper chamber in DMEM medium free of FBS but containing L-securinine at concentrations of 0 (control), 2.5, 5, and 10 μM, and the lower chamber was filled with medium supplemented with 20% FBS as a chemoattractant. After incubation at 37°C for 48 h, the cells remaining on the surface of the upper chamber were cleaned off by a cotton swab, while the migrated or invaded cells to the lower surface of the chamber were fixed in 95% ethanol for 5 min and stained with 0.2% crystal violet in 10% ethanol for 3 min. Six random microscopic fields of invasive or migratory cells per well were counted under a microscope at a magnification of ×200 to determine the cell numbers, and the data were calculated as percentage of the control group. Each experiment was performed in triplicate.

### Total protein extraction and western blot analysis

After treatment, cells were washed twice with PBS and total protein extraction from the cultured cells was performed as described previously [18]. The protein content was determined by Bradford method and equalized before loading. The protein extracts (20 μg) were separated by 10% SDS-PAGE gels and then transferred to a nitrocellulose membrane. After blocking with 5% nonfat milk for 1 h, the membranes were incubated with specific primary antibodies of Bcl-2 (1:2000), Bax (1:1000), cleaved caspase-3 (1:1000), cleaved caspase-8 (1:1000), cleaved caspase-9 (1:1000), MMP-2 (1:500), MMP-9 (1:500), AGTR1 (1:1000), p-MEK1/2 (1:1000), ERK1/2 (1:1000), p-ERK1/2 (1:1000), PAX2 (1:1000), p-PAX2 (1:1000), VEGF (1:1000), STAT3 (1:1000), p- STAT3 (1:1000), and β-actin (1:200) overnight 4°C. Subsequently, the membranes were incubated with the appropriate horseradish peroxidase (HRP)-conjugated secondary antibodies (1:5,000) 1 h at room temperature. The blots were developed with an ECL chemiluminescence reagent and relative protein expression levels were normalized to the β–actin reference by comparing the density of each band.

### Statistical analysis

All values were presented as mean ± S.D. of three independent experiments. Statistically significant differences were performed using the two-tailed Student’s *t*-test or one-way ANOVA, and differences were considered significant when *P* value less than 0.05.

## Results

### L-securinine inhibits the proliferation of prostate cancer cells

To determine the cytotoxicity of L-securinine on prostate cancer cells, two kinds of cell lines (androgen-independent DU145 cells and androgen-dependent LNCaP cells) were treated with L-securinine (2.5, 5, and 10 μM) for 24, 48, and 72 h, and MTT assay was performed to measure the cells’ growth. As demonstrated in Figure 2, treatment with 2.5, 5, and 10 μM of L-securinine resulted in a stronger inhibitory effect on cell viability of androgen-independent DU145 cells. Of note, there were significant differences between the treatment groups and the control group at each time point for DU145 cell line, especially when the treatment time exceeded 48 h (*P*<0.05 or *P*<0.01). At the end of 48 h, cell viability decreased from 100% in control cells to 71.99 ± 7.26, 54.28 ± 5.28, and 34.48 ± 5.84% for DU145 cells, respectively, which was close to those at 72 h. However, no significant inhibitory effect of can be observed in androgen-dependent LNCaP cells after 24 and 48 h exposure of L-securinine at any concentrations (*P*>0.05), and only a significant inhibitory effect occurred at the high concentration of L-securinine (10 μM) after 72 h treatment compared with the control cells (*P*<0.05). These findings confirmed that androgen-independent DU145 prostate cancer cells were more sensitive to L-securinine treatment than androgen-dependent LNCaP cells. In the next study, we used DU145 cells as model cells to study the antitumor mechanism of L-securinine.

**Figure 2:** Effect of L-securinine on the cell viability of androgen-independent DU145 cells and androgen-dependent LNCaP cells (**A**) Effect of L-securinine (2.5, 5, and 10 μM) on the cell viability of DU145 cells at 24, 48, and 72 h; (**B**) effect of L-securinine (2.5, 5, and 10 μM) on the cell viability of LNCaP cells at 24, 48, and 72 h. Results are expressed as the percentage of the cell viability relative to the viability of control and data are presented as the mean ± S.D. of three independent experiments (*n*=3). Significant at *P<0.05; **P<0.01 compared with control cells.

### L-securinine induces the apoptosis of prostate cancer cells

To examine whether the cell–growth suppressive effect of L-securinine on androgen-independent DU145 prostate cancer cells is mediated by apoptosis, nuclear Hoechst 33258 staining was employed to verify the morphological changes in the apoptotic cells. As indicated in Figure 3A, L-securinine–treated cells exhibited typical apoptotic morphological features such as bright blue condensed chromatin or fragmented nuclei. By contrast, the untreated cell nuclei displayed homogeneous and round nuclei with less intense staining.

**Figure 3:** Effect of L-securinine on the apoptosis of DU145 cells (**A**) Morphological analysis of the nucleus was evaluated in DU145 cells by Hoechst 33258 staining; (**B**) analysis of L-securinine-induced apoptosis by flow cytometry assay using Annexin V-FITC/PI double-staining; (**C**) quantitation of flow cytometry analysis. Data are presented as the mean ± S.D. of three independent experiments (*n*=3). Significant at * *P*<0.05; **P<0.01 compared with control cells

Next, we further quantitated the apoptosis of L-securinine-treated DU145 cells by flow cytometry assay using Annexin V-FITC/ PI dual-labeling technique. As expected, L-securinine was found to induce apoptosis in DU145 cells in a concentration-dependent manner (shown in Figure 3B,C). The percentage of apoptotic cells were increased by L-securinine from 8.5% in control cells to 39.53% at 2.5 μM, 51.62% at 5 μM, and 64.23% at 10 μM, respectively (*P*<0.05 or *P*<0.01). These results suggest that L-securinine effectively promoted apoptosis of DU145 cells in a dose–dependent manner.

### L-securinine inhibits the invasion and migration of SGC7901 cells

Because cell invasion and migration are common features in the process of tumor metastasis, Transwell assay coated with or without Matrigel were conducted to detect the influences of L-securinine on the invasive and migratory ability of DU145 cells *in vitro*, respectively. Compared with the control, L-securinine displayed a remarked dose-dependent inhibitory effect on the cell number of DU145 cells that invaded or migrated to the lower chamber (Figure 4D, *P*<0.01 or *P*<0.001). The invasion rate dropped from 100% in control cells to 60.66, 31.58, and 23.85% in DU145 cells after exposure of 2.5, 5, and 10 μM of L-securinine, respectively. Similar results were observed *in vitro* migration assays, as showed by the decreased number of 82.01, 46.13, and 22.42% of DU145 cells in the lower chamber in response to 2.5, 5, and 10 μM of L-securinine treatment, respectively. Both *in vitro* invasion and migration assays suggested that L-securinine had the potential to inhibit prostate cancer metastasis.

**Figure 4:** Effect of L-securinine on the metastasis of DU145 cells (**A**) Effects of L-securinine (2.5, 5, and 10 μM) on cell invasion of DU145cells; (**B**) histogram showing the Transwell invasion assays of DU145 cells in each group; (**C**) effects of L-securinine (2.5, 5, and 10 μM) on cell migration of DU145 cells; (**D**) histogram illustrating the Transwell migration assays of DU145 cells in each group. Data are presented as the mean ± S.D. of three independent experiments (*n*=3). Significant at ** *P*<0.01; ***P<0.001 compared with control cells.

### L-securinine regulates the expression of cancer apoptosis-associated proteins

To further delineate the mechanism by which L-securinine induced apoptosis on DU145 cells, the expression of apoptosis-associated proteins, such as Bax, Bcl-2, cleaved caspase-3, cleaved caspase-8, cleaved caspase-9, and cytosolic cytochrome c, was examined by western blot assay. As shown in Figure 5, after treatment of L-securinine, it was found that the expression of pro–apoptotic Bax protein was increased, while the expression of antiapoptotic Bcl-2 protein appeared to be markedly decreased in a dose-dependent manner in DU145 cells and the differences were statistically significant compared with the control group (*P*<0.05, *P*<0.01, or *P*<0.001). Moreover, a significant increase in cleaved caspase-9 and cleaved caspase-3 were detectable in DU145 cells following L-securinine treatment (2.5, 5, and 10 μM), followed by the cleavage of poly-(ADP-ribose)-polymerase (PARP), a known substrate of caspase-3. However, cleaved caspase-8 kept unchanged during the incubation with L-securinine treatment for 48 h (*P*>0.05). In addition, a dose-dependent release of cytochrome c into the cytoplasm from the mitochondria was significantly promoted in L-securinine-treated DU145 cells with relative to the untreated cells (*P*<0.05 or *P*<0.001). These data indicate that L-securinine-induced apoptosis in DU145 cells is partly mediated through the mitochondrial pathway.

**Figure 5:** Effects of L-securinine (2.5, 5, and 10 μM) on the protein expression of Bax, Bcl-2, cleaved caspase-9, cleaved caspase-8, cleaved caspase-3, cytosolic cytochrome c, and cleaved PARP in DU145 cells Data are presented as the mean ± S.D. of three independent experiments (*n*=3). Significant at *P<0.05; **P<0.01; ***P<0.001 compared with control cells.

### L-securinine suppresses the expression of androgen-independent prostate cancer -associated proteins

Moreover, we also investigated the expression of androgen-independent prostate cancer-associated proteins including MMP-9, MMP-2, AGTR1, MEK1/2, p-MEK1/2, ERK1/2, p-ERK1/2, STAT3, p-STAT3, PAX2, p-PAX2, and VEGF, which are also consensually considered to be related with cell proliferation, migration, and invasion of prostate cancer cells. As Figure 6 illustrated, in untreated cancer cells, the protein expression of MMP-2, MMP-9, AGTR1, PAX2, p-MEK1/2, p-ERK1/2, p-STAT3, and VEGF showed a higher expression level than those in L-securinine-treated cells. Following 48 h treatment of DU145 cells with L-securinine (2.5, 5, and 10 μM) dramatically decreased these protein expressions in a dose-dependent manner, whereas the protein expression of ERK1/2, MEK1/2, and STAT3 remain almost unchanged before and after L-securinine treatment. Collectively, these results supported the idea that L-securinine suppressed the growth and metastasis of androgen-independent DU145 cells via blocking AGTR1, as well as inhibiting the activation of their downstream target signal pathway of MEK1/2, ERK1/2, STAT3, and PAX2.

**Figure 6:** Effects of L-securinine (2.5, 5, and 10 μM) on the protein expression of MMP-9, MMP-2, AGTR1, MEK1/2, p-MEK1/2, ERK1/2, p-ERK1/2, STAT3, p-STAT3, PAX2, p-PAX2, and VEGF in DU145 cells Data are presented as the mean ± S.D. of three independent experiments (*n*=3). Significant at *P<0.05; **P<0.01; ***P<0.001 compared with control cells.

## Discussion and conclusion

The objectives of the present study were to demonstrate how L-securinine induces apoptosis and inhibits metastasis in androgen-independent DU145 cell line, and to decipher the mechanisms and identify the key signaling molecules responsible for this effect. Uncontrolled cell proliferation is a hallmark of tumorigenesis and inhibiting proliferation can enable growth arrest in tumor cells [19]. As determined by MTT assay, L-securinine (2.5, 5, and 10 μM) treatment resulted in a dose and time-dependent inhibitory effect on the proliferation of androgen-independent DU145 cells, especially beyond 48 h. Whereas, no obvious cell growth inhibitory effect was detected in androgen-dependent LNCaP cells, except at the concentration of 10 μM and after 72 h incubation. This sensitivity difference suggested that L-securinine is prone to suppress androgen-independent DU145 cell line. As we know, cell apoptosis, a programmed cell death process, is believed to be one of the major parameters that incurred growth loss of cancer cell [20]. To further determine if this growth inhibition by L-securinine was associated with the apoptosis induction, we used Hoechst 33258 staining to examine morphological change in DU145 cells and then quantitated the percentage of apoptotic cells with flow cytometry assay using Annexin V-FITC/ PI dual-labeling. After 48 of treatment in the presence of L-securinine (2.5, 5, and 10 μM), distinct apoptotic morphological abnormalities including cell shrinkage, chromatin condensation, and formation of apoptotic bodies were observed with Hoechst 33258 staining by fluorescence microscope, compared with the control. FACS analysis showed that L-securinine (2.5, 5, and 10 μM) induced apoptosis in DU145 cells and the apoptotic cell number increased as the dose increased. Clearly, an agent like L-securinine, which could efficiently inhibit the proliferation and induce apoptosis of cancer cells, would be a hopeful alternative medicine to suppress cancer progression and thus could reduce mortality.

Tumor metastasis is the spread of cancer cells from primary neoplasm to a distant location via blood or lymph vessels [21], and ultimately leads to a high mortality rate and poor prognosis [22]. This process requires tumor cell adhesion, migration, and enzymatic degradation of the extracellular matrix and basement membrane [23]. Hence, blockading of invasion and migration ability of cancer cells would prolong cancer patients’ lifetime. As anticipated, the results of Transwell assay showed that the migratory and invasive abilities of the DU145 cells were dose-dependently suppressed by L-securinine treatment for 48 h compared with the control cells.

To the best of our knowledge, apoptotic cell death is strictly controlled by certain internal or external signals. Presently, two major pathways leading to apoptotic cell death have been revealed. One is the death-receptor-induced extrinsic apoptosis pathway where the cell surface receptors interact with their ligands, followed by the cascade of upstream caspase-8 [24], and the other is the mitochondrial-mediated intrinsic apoptosis pathway which involves the participation of the antiapoptotic and proapoptotic members of the Bcl-2 family, cytochrome c release from the mitochondria and activation of caspase-9 [25]. Caspase-8 is the key initiator of death receptor-mediated extrinsic apoptosis, whereas caspase-9 is regarded as the canonical caspase in the intrinsic mitochondrial pathway [26]. To investigate the pathways involved, the protein expression of Bax, Bcl-2, cleaved caspase-9, cleaved caspase-8, cleaved caspase-3, cytosolic cytochrome c, and cleaved PARP were determined in DU145 cells. Accordingly, L-securinine treatment decreased the expression of Bcl-2 protein and increased the level of Bax, cleaved caspase-9, cleaved caspase-3, cytosolic cytochrome c, and cleaved PARP protein expression. In contrast, cleaved caspase-8 remained unchanged. These results together suggest that the mitochondrial, but not the death receptor pathway, is involved in L-securinine-induced apoptosis in DU145 cells.

Apart from the involvement of mitochondrial intrinsic apoptosis pathway in L-securinine-induced apoptotic cell death, there must be some other exclusive regulatory molecules responsible for this antitumor activity toward androgen-independent prostate cancer DU145 cells. It is well known that the proteolysis of the basement membrane is predominantly achieved by MMPs family, such as MMP-2 and MMP-9, which are capable of degrading type IV collagen, a major component of the basement membrane [27]. Higher levels of MMP-2 and MMP-9 were reported to be associated with the metastasis in many malignant tumor cells including androgen-independent prostate cancer [28]. Moreover, various MMPs are also necessary for releasing proangiogenic factors like VEGF [29], which acts on endothelial cells to induce cell migration and proliferation [30]. It has been verified that VEGF has a positive regulation with MMP-2 and MMP-9 activity in DU145 human prostate cancer cells [31]. Here in our study, our data have revealed that L-securinine treatment led to inhibited expression of MMP-2 and MMP-9 and concurrent reduction in the levels of VEGF. As noted in another important reference by Bose et al [32], inactivation of AGTR1/MEK/ERK/STAT3/PAX2 pathway resulted in a sharp decrease of cell viability of DU145cells. In line with this mechanism, a similar decrease in the protein expression of AGTR1, p-MEK1/2, p-ERK1/2, p-STAT3, PAX2, and p-PAX2, was observed in L-securinine stimulated DU145 cells, although ERK1/2, MEK1/2, and STAT3 protein expression kept unchanged.

Along with these data, our present research demonstrated that L-securinine is effective in inhibiting proliferation and metastasis of androgen-independent DU145 cells *in vitro*, suggesting L-securinine may be a leading candidate in developing preventive agents for the treatment of AIPC.

## Availability of data and materials

The analyzed datasets generated during the study are available from the corresponding author on reasonable request. All authors have read and approved the final manuscript.

## Abbreviations

AIPC: androgen-independent prostate cancer
FBS: fetal bovine serum
HRP: horseradish peroxidase
FITC: fluorescein isothiocyanate
PI: propidium iodide
PARP: poly-(adenosine diphosphate ribose) polymerase
